This article has been retracted.

# Blockchain and IPFS Integrated Framework in Bilevel Fog-Cloud Network for Security and Privacy of IoMT Devices

**DOI:** 10.1155/2021/7727685

**Published:** 2021-12-07

**Authors:** Abolfazl Mehbodniya, Rahul Neware, Sonali Vyas, M. Ranjith Kumar, Peter Ngulube, Samrat Ray

**Affiliations:** ^1^Department of Electronics and Communication Engineering, Kuwait College of Science and Technology (KCST), Doha Area, Kuwait; ^2^Department of Computing, Mathematics and Physics, Høgskulen på Vestlandet, Bergen, Norway; ^3^University of Petroleum and Energy Studies, Dehradun, India; ^4^Department of Mathematics, Amrita School of Engineering, Amrita Vishwa Vidyapeetham, Chennai, India; ^5^Malawi University of Science and Technology, Malawi; ^6^The Institute of Industrial Management, Economics and Trade, Peter the Great Saint Petersburg Polytechnic University, Russia

## Abstract

Internet of Medical Things (IoMT) has emerged as an integral part of the smart health monitoring system in the present world. The smart health monitoring deals with not only for emergency and hospital services but also for maintaining a healthy lifestyle. The industry 5.0 and 5/6G has allowed the development of cost-efficient sensors and devices which can collect a wide range of human biological data and transfer it through wireless network communication in real time. This led to real-time monitoring of patient data through multiple IoMT devices from remote locations. The IoMT network registers a large number of patients and devices every day, along with the generation of huge amount of big data or health data. This patient data should retain data privacy and data security on the IoMT network to avoid any misuse. To attain such data security and privacy of the patient and IoMT devices, a three-level/tier network integrated with blockchain and interplanetary file system (IPFS) has been proposed. The proposed network is making the best use of IPFS and blockchain technology for security and data exchange in a three-level healthcare network. The present framework has been evaluated for various network activities for validating the scalability of the network. The network was found to be efficient in handling complex data with the capability of scalability.

## 1. Introduction

The present world with a fast-growing global economy and the latest advancements in technology has led to the industry 4.0 revolution [1]. The outbreak of COVID-19 and many other chronic diseases has been observed in the last decade. The population explosion and outbreaking of chronic and other diseases have led to deterring health issues [2]. In the present day, the prevention and maintaining a healthy lifestyle have become essential for long and healthy living. The increasing number of patients and lack of medical services can lead to daunting circumstances in any state or country. Thus, the integration of medical services and information technology has become an essential need [3]. The industry 5.0 and 5G has led to the development of cost-efficient sensors for medical services, which eventually led to the emergence of Internet of Medical Things (IoMT) [4]. In the present world scenario, telemedicine, smart/remote healthcare has gathered special attention in disease prevention and monitoring/maintaining a daily healthy lifestyle. The schematic of IoMT has been shown in Figure 1.

With industry 5.0, revolution and 5G technology have made possible the use of sensors and devices which can sense data and transfer it wirelessly to the remote cloud by wireless communication network [5]. The cost-efficient sensors have led to the emergence of wearable devices and gadgets which can monitor various essentials and human body vitals such as blood pressure, saturation level, pulse rate, breathing rate, measure of distance, and elevation covered [6]. Amount of deep sleep taken and number of times certain activities are done. To enhance the healthy lifestyle, these gadgets and devices are connected to smart mobile phones which keep reminders of medicine, physical activities, deep breathing sessions, important medical meetings, etc. [7]. These sensors and devices generate huge E-health data that need AI and deep learning technologies for proper interpretation along with cloud computing and storage for efficient data management and data communication [8, 9]. The security of this health data is necessary. The prevention of falling in wrong hands may lead to misuse of data for personal gain. The misuse of E-health data can be done by any pharmaceutical companies or certain hospitals for creating a monopoly of services and thus induce gains [10]. To avoid such circumstances, data security and privacy is the top priority. Many data security frameworks and models have been presented for E-health and IoMT data [11]. In recent times, blockchain has gained trust in data privacy and security domain as compared to other technologies [12]. Decentralized structure of the blockchain framework has been the main advantage. Another decentralized structure is also known as an interplanetary file system (IPFS), which allows data exchange across the network in a more secure way than the conventional central server system by peer-to-peer (P2P) communication. The main advantage of using IPFS is that the user on the network uses public gateways instead of installing IPFS clients. IPFS can be used for mirroring websites, speeding up the secure network without creating any nodes, to name a few. The present work has been focused and developed a block-chained integrated multitier network for real-time monitoring of E-health data with the main purpose of enhancing and maintaining a healthy lifestyle [13]. The proposed framework has been tested for scalability and network efficiency in terms of data transfer and data preservation. For the development of the proposed model, the author has done a thorough literature survey of closely related works and has been presented in the next section.

## 2. Related Work

In recent studies, Deebak et al. [14] have device single user sign-in (SUSI) mechanism for the protection of multimedia data using the public key and encryption-decryption method in Remote Medical Point of Care (RM-PoC). The simulation studies have shown the higher efficiency in data computation and data transmission processes.

Another parallel work of Selvaraj et al. [15] has presented an extended coverage global system for mobile communications. GSM IoT protocol-based framework. The proposed framework was integrated with the wide mouth frog protocol for secure data transmission and prevents insider attacks, DDoS, and other intermediate attacks. The network model was successful in preventing inside and intermediate DDoS attacks while maintaining high data integrity and low latency and high scalability.

Bharti et al. [16] presented a particle swarm optimization-based directed weighted complex network using a genetic algorithm. The proposed model was used to solve the optimal key-based medical image encryption of sensitive and confidential image data. The proposed model was successful and efficient in encrypting and decrypting medical image data while maintaining the speed of convergence without loss of diversity.

Similarly, researcher Islam et al. [17] made a smart healthcare monitoring system to monitor real-time patient health data and room condition. The developed system was successful in monitoring patent and room conditions along with transfer of data to the healthcare professional via a portal.

Similarly, Maragathavalli et al. [18] have worked on modified decoy technique for securing medical big data. A third party used authentication agreement protocol for medical data of the patient stored in cloud storage. The proposed framework is helpful in identifying hacker IP address, date, and time stamps. The modified technique has increased the network throughput by 20% and decreased computation technique.

Lv and Piccialli integrated k-anonymity and differential privacy [19]. The simulation studies of the proposed model along with comparative analysis of the proposed and existing models. Analysis of the hybrid algorithm has shown a reduced risk of privacy information loss for medical data. A biometric-based security framework has been developed by Pirbhulal et al.; the proposed model was able to record real-time ECG and heartbeat-related data from wearable devices. The proposed model was found to work more efficiently compared to its competitive model in terms of computational cost and time.

Selvakanmani and Sumathi [20] have proposed the blockchain and smart contract-based framework for cloud-edge computing in the healthcare system, thus providing data privacy, security, latency, cost-effective storage, and data availability.

After closer analysis of the related work and other models [4, 20–23], we have found that most of the security networks are centralized in nature which rely on third-party sources for security and data exchange. The healthcare system is spread across heterogeneous platforms and devices, which enforces the developer to think about a decentralized framework for easy data exchange with complete security and privacy. The main drawback of a centralized network is the single point of failure by a single point of attack by unauthorized devices and users. Moreover, cloud computing has become indispensable and the accessibility of cloud data is an on-demand service which is provided by a third-party source [10]. Most of the proposed healthcare systems are not able to exploit both IPFS and blockchain technologies. There is a strong demand of decentralized system for accessing the cloud services and data which are provided best by blockchain and smart contract technology. Most of the networks used blockchain only at one level, while the breach of data at the lower level is always possible. The present work has implemented the hybrid blockchain at 3 levels network of edge, fog, and cloud level framework which will be useful in E-health and medical communication services. The proposed model working methodology and architect is presented in Section 3, which describes the parallel integration of IPFS and blockchain in three-level frameworks for handling healthcare data, followed by the results and discussion in Section 4 where the efficiency of the proposed network has been compared by varying the number of peers and the size of data transaction along with the role of IPFS and blockchain in the present framework. The conclusion and future scope are briefed in Section 5.

## 3. Methodology

In the proposed framework and a decentralized structure made for the authentication of medical devices, sensors as well as storage of data which can easily be compromised in security and privacy in IoMT enabled healthcare. The proposed model works in two segments. The first segment is responsible for authentication and authorization of patient registration and medical devices. The second segment disseminates the patient and device information in the integrated blockchain network. These two segments are directly integrated in the fog network. The information is then exchanged between fog and cloud using the hybrid blockchain framework. The schematic of the proposed framework has been presented in Figure 2.

Hybrid blockchain is implemented to reduce the attack probability drastically as the number of blocks in the chain increases. For *n* number of block differences between the actual and attacker blockchain, the chance of successful attack is given by normal distribution and given by the equation.

(1) $$\begin{array}{c} P_{n}=1-\overset{n}{\underset{k=0}{\sum }}\frac{\lambda^{k}e^{-\lambda }}{k!}\left\{1-\left(\frac{q}{p}\right)\right\},\;\lambda =n\frac{q}{p}. \end{array}$$

In Equation (1), *q* represents the computational resources under the attacker command and *p* is equal to the fraction of the remaining resources in the network. However, in hybrid blockchain, the attacker chances are calculated by

(2) $$\begin{array}{c} P_{n}=1-\overset{n}{\underset{k=0}{\sum }}\frac{\lambda^{k}e^{-\lambda }}{k!}\left\{1-\overset{n-k}{\underset{m-1}{\prod }}\left(\frac{q}{p}\right)\right\},\;\lambda =\overset{n}{\underset{m=1}{\sum }}\frac{q}{p}. \end{array}$$

In Equation (2), the odd values of *q*/*p* represent the resources and the even value represents the ratio of other resources. The *n* here represents the number of blocks the recipient of a new transaction required to wait to prevent the attacker's success.

IPFS will confirm the simultaneous authentication of the patients and their corresponding medical devices. This will lead to a secure system of storage in IoMT devices. IPFS cluster nodes synchronize the data and information along with authorization and authentication of the medical devices. It also plays an important role in blockchain activities such as transaction mapping, block creation, and communication with smart contract to name a few.

Communication between the cluster nodes, IoMT devices, blockchain, fog, and cloud is essential to understand. The medical devices first communicate with IPFS cluster nodes for registration of the patient and the respective medical devices. After registration, a few lists of authorized services and accesses are generated and transferred to the fog network using a private blockchain. The fog network is responsible for partial or semiprocessing of the data depending on the requirement. The semiprocessed data is then sent to the cloud via a public blockchain where high computational resources are available for processing the IoMT data. The useful and via information obtained from the processed is then shared with the IoMT devices. Smart contracts for both public and private blockchains ensure the secure and private automation of the data exchange process among the devices of patients, healthcare professionals, and doctors.

For device authentication, the IoMT device interacts with IPFS cluster nodes by a smart contract which registers the IoMT device first. IPFS nodes will then send the registration detail data to the blockchain. Consequently, a block is generated with the transaction details provided by the IPFS node. The generated block is then deployed in the blockchain network after successful registration. Whenever the device interacts with the blockchain network, the interaction is first authorized by the smart contract details generated earlier by the IPFS cluster node. Once the smart contract is deployed to any IoMT device, it becomes automatically secure. The other defaulter blocks cannot be allowed to interact with the blockchain as they are not registered in the distributed ledger on the blockchain. Based on the various available algorithms available, the modified LMDS algorithm is used for the generation of public and private keys for IoMT devices. Once the IoMT devices and the respective patient are registered with the patient ID in the network, then the IoMT devices are identified and authorized to access the services available on the fog and cloud network.

The patient registration, patient ID generation, and linking of medical devices are done as per the proposed algorithm. Similarly, algorithms are proposed for the medical device registration and linking of patient ID with device id.

After successful generation of patient ID, the device is then registered in the same manner, as shown in Algorithm 2.

Once the valid patient ID and device ID are generated and updated in the IPFS database and blockchain, then linking/mapping of the patient and device is done using the following algorithm.

After integration of the IoMT device and patient ID, the block is generated and added to the blockchain. And a list of accessible services is generated. The details of this information are stored in the blockchain at the fog network.

## 4. Results and Discussion

The proposed framework has been evaluated for data integrity, confidentiality, nonrepudiation, parallel identification, and parallel authentication using node.js solidity version 0.10.42. The smart contracts were allowed to directly interact with the application interface for device verification and storage of address. The experiments were carried out on an intel Xenon silver 4114 CPU with 64 GB RAM and 1 TB HD.

The following Figure 3 shows the energy consumption of the operations in the proposed framework. 93% of the energy consumption was made in permission access, revoke permission, and removing patient activities, followed by 6% energy consumption in contract deployment and less than 1% in adding agents.

A similar trend was observed in the time consumption network activities (Figure 3). A major chunk of time was consumed in permission access, revoke access, and removing patients (up to 80%) whereas 16% and 13% were consumed by deploying contracts and adding agent, respectively. The activities like permission access, revoke access, and removing patient require to access the network at blockchain integrated fog and cloud level for data transactions. The processing of complex data generated by blockchain requests time and energy for processing; thus, it takes more time and energy as compared to other activities. Registration of IoMT devices on the peer network is necessary to prevent the vulnerability of the device. The time required to complete registration is presented in Figure 4.

It is observed that the registration time per peer for increasing number of peers is decreasing. The drop of 2 milliseconds is observed from 5.5 milliseconds for a single peer to 3.5 milliseconds per peer for 25 peers' registration. The drop of time is almost 35%. The proposed algorithm allows the parallel registration of peers and thus improves the registration execution time. The present framework allows parallel processing of peers, which reduces the execution time.

For uploading of the file has been done by varying the number of transactions and presented in Figure 5, one file is converted into data packets of 40, 80, 160, and 320 packets. The time for uploading various data packets per peer for 25 peers has been shown in Figure 5. It has been found that with decreasing the size of data packet, the uploading time increases per peer. However, the uploading time per peer decreases with increasing number of peers. The least time of upload has been observed in for large data size packet for 25 peers. This proposed framework allows larger file transactions on a large number of peers with higher speed.

Execution time of nonrepudiation for different data packet transactions per peer is presented in Figure 6. The nonrepudiation increases per peer with decreasing the size of data packet transaction. With increasing number of peers, the data transaction per peer first decreases sharply for 10 peers and then increases for 15 peers, followed by a decreasing trend for 20 and 25 peers.

Execution of block mining has been calculated for various transaction sizes per peer as shown in Figure 7. It was found that with decreasing size of data transaction, the block mining execution time per peer increases. Whereas with increasing number of peers, the trend was not the same. With increasing number of peers, the mining execution time per peer firstly decreases for 10 peers and then increases slightly for 15 peers, followed by a decreasing trend for 20 and 25 peers.

However, the block creation time for various data sizes, transactions, and number of peers was the same (Figure 8). With increasing number of peers, the block creation time per peer was found to be decreasing. On the other hand, with decreasing the size of transaction, the mining time increases drastically.

The final step of contract deployment was also evaluated and has been presented in Figure 9. It has been found that, with decreasing size of data transaction, the contract deployment time per peer increases. However, on the other hand, the contract deployment time per peer decreases with increasing number of peers on the network.

The proposed network has shown the comparative better performance with maximum number of peers and small data packet transaction as compared to small number of peers and large data packet transaction. The use of IPFS leads to low latency and less energy consumption due to its inherent nature. IPFS allows data replication across multiple nodes, thus facilitating collaborative efforts for data storage. The consolidated data of the results has been presented in Table 1.

## 5. Conclusion and Future Scope

The present work shows the successful implementation of a 3-layer framework for real-time monitoring of patient data. The proposed mode was able to identify and authenticate the peers and devices along with verification of nonrepudiation of transactions made by the medical devices. Prevention of proof Sybil replay and substitution attack. Owing to certain advantages such as blockchain-based decentralized network which poses lesser security risk compared to the centralized networks, the registration-based model for device and patient mapping does not allow the unregistered patient or device to access the data and services, thus preventing data loss and data misuse. This also allows the patients and users the customized access of services and data, thus making the network more secure. The use of blockchain at fog and edge level makes the double-layer security. The optimized resource allocation at fog and edge level makes the network more efficient in terms of data processing, data transfer, and relay of information. The present model has shown scalability; thus, the future work comprises of implementation of the model for trauma services where real-time monitoring is critical.

## Figures and Tables

**Figure 1:** IoMT and its benefits.

**Figure 2:** The proposed framework for IoMT and patient registration.

**Figure 3:** Energy and time consumption for various IoT activities.

**Figure 4:** Registration time of IoT device peer for various numbers of peers.

**Figure 5:** Execution time of uploading for various sizes of file transactions (Txn) per peer for various numbers of peers.

**Figure 6:** Execution time for nonrepudiation of Txn per peer for various numbers of peers.

**Figure 7:** Time required for block mining per peer for various numbers of peers.

**Figure 8:** Time required for block creation varying number of peer and transactions.

**Figure 9:** Time required for contract deployment for varying number of Txn and peers.

**Algorithm 1:** Patient registration.

**Algorithm 2:** Device registration.

**Algorithm 3:** Device authentication in IoMT blockchain.

**(a):** 

Execution time (seconds) in upload of data per peer for varying transactions (Txn)				
Number of peers	For 40 Txn	For 80 Txn	For 160 Txn	For 320 Txn
5	0.149	0.167	0.186	0.197
10	0.086	0.097	0.102	0.110
15	0.060	0.065	0.070	0.100
20	0.046	0.061	0.063	0.091
25	0.037	0.061	0.066	0.092

**(b):** 

Execution time analysis of nonrepudiation per peer for varying transactions (Txn)				
Number of peers	For 40 Txn	For 80 Txn	For 160 Txn	For 320 Txn
5	1.639	3.881	8.059	18.510
10	0.890	2.534	4.178	10.374
15	1.640	3.182	6.665	13.534
20	1.118	2.684	5.559	10.598
25	1.193	2.625	6.210	10.629

**(c):** 

Execution time for block mining per peer for varying transactions (Txn)				
Number of peers	For 40 Txn	For 80 Txn	For 160 Txn	For 320 Txn
5	2.167	4.064	7.985	16.712
10	1.082	2.540	4.436	9.245
15	1.610	3.296	6.540	12.275
20	1.205	2.661	5.476	9.775
25	1.217	2.634	6.151	7.795

**(d):** 

Execution time for block creation per peer for varying transactions (Txn)				
Number of peers	For 40 Txn	For 80 Txn	For 160 Txn	For 320 Txn
5	2.834	5.522	8.358	18.805
10	2.910	5.223	4.402	10.447
15	2.388	3.781	6.766	13.781
20	1.455	3.619	5.783	10.708
25	0.388	0.865	6.417	10.686

**(e):** 

Execution time for block access per peer for varying transactions (Txn)				
Number of peers	For 40 Txn	For 80 Txn	For 160 Txn	For 320 Txn
5	2.121	3.939	8.333	18.939
10	2.575	2.878	4.318	10.606
15	2.373	3.484	6.767	13.888
20	1.401	2.878	5.757	10.871
25	0.393	2.757	6.484	10.909

**(f):** 

Execution time contract deployment per peer for varying transactions (Txn)				
Number of peers	For 40 Txn	For 80 Txn	For 160 Txn	For 320 Txn
5	2.236	3.947	8.552	18.684
10	1.381	2.763	4.602	9.342
15	1.798	3.333	6.842	12.631
20	1.414	2.960	5.756	10.263
25	1.473	2.842	6.421	9.105

## Data Availability

The data used to support the findings of this study are available from the corresponding author upon request.
